# Application of Sandplay Therapy in the Mental Health Education of Vocational College Students

This article has been retracted.

**DOI:** 10.1155/2022/6141326

**Published:** 2022-06-29

**Authors:** Xiaojing Xu, Yanhua Zhang, Libin Liu

**Affiliations:** Shaanxi Business College, China

## Abstract

**Objective:**

To analyze the application and effect of sandplay therapy in higher vocational students' mental health.

**Method:**

350 sophomores of 2019 in a higher vocational college were randomly selected, and 72 subjects of depressed students (SAS ≥ 50) were selected from 350 sophomores and randomly divided into the intervention group and the control group, each group 9, preparing one set of chamber equipment, adopting the same group before and after test experiment design. The intervention group was, respectively, given 8 individual box court game tutoring, once a week for each person. The control group did not intervene. By comparing the intervention group with the control group, the intervention effect of sandplay therapy on anxiety of experimental group members was investigated.

**Results:**

Among 350 respondents, 72 had SAS scores ≥ 50, and the incidence of anxiety symptoms was 20.57%. Since there was only 1 case with SAS score ≥ 70, it was incorporated into the group with SAS score ranging from 60 to 59. After treatment, SAS scores of students with mild to moderate anxiety in the intervention group decreased, and the difference was statistically significant. The difference before and after control group was not statistically significant. After sandplay therapy, the differences in SAS scores between the intervention group and the control group were found to be statistically significant for both mild and moderate anxiety.

**Conclusion:**

Sandplay therapy in the higher vocational college students' mental health education could promote the mental health of students, and it effectively improves students' psychological quality.

## 1. Introduction

With the changes of learning pressure and social environment in colleges and universities, the psychological diseases of college students show an increasing trend (depression, anxiety disorder, bipolar disorder, etc.) [1, 2]. Sandplay therapy is a kind of psychotherapy in which an individual, accompanied by the therapist, selects toys from the toy shelf freely and performs self-expression in a special box filled with fine sand [3]. In 1954, combining Jung's analytical psychology and projection techniques, Dore M. Kalff developed Lowenfeld's “The World Technique,” it was introduced to Japan by a Japanese clinical psychologist, and Zhang Risheng introduced it to China in 1998 [4]. Sandplay therapy creates “free and protected spaces” through sand, water, and toys, providing visitors with the possibility of expressing unintentional processes [5]. The visitors solve their personality problem on this basis, and the symptoms are also eliminated [6], thereby improving or eliminating psychological disorders such as anxiety and depression [7]. The sandplay therapy itself is nonverbal and nondirective. The client expresses his emotions in the chamber consciously or unconsciously. In the face of the sandplay works created by himself, through sharing and analysis with the therapist, the visitor will have awareness of his own cognition and emotions, so as to improve or eliminate his anxiety, depression, and other psychological disorders [8, 9]. At the initial stage of group sandplay therapy intervention, trauma themes such as division and hostility often appear. After the implementation of group sandplay therapy intervention, the sensitivity level of students' interpersonal relationship has decreased significantly, and their personal sense of discomfort and inferiority have improved. Group sandplay therapy shows a certain curative effect. Sandplay therapy is one of the important methods of emotional management education [10, 11]. Sandplay therapy can help college students find their own problems, rebuild their cognition, and vent their emotions [12]. The mental health education of higher vocational students is of particularity. Its treatment targets are mainly growing and developing college students. Most of their psychological problems are developmental problems. Therefore, sandplay therapy can be used in college mental health education. This study selected 350 sophomore depressed students from our school to conduct a sandplay analysis.

## 2. Materials and Methods

### 2.1. Research Object

350 sophomores of 2019 in a higher vocational college were randomly selected, and 72 subjects of depressed students (SAS ≥ 50) were selected from 350. Among them, there were 40 girls and 32 boys, aged from 20 to 22 years. The average age of the subjects was 21.24 years. The subjects were randomly divided into the intervention group and control group, each group 9. Basic information of research object is shown in Table 1:

### 2.2. Methods

#### 2.2.1. Equipment Preparation

One set of box court equipment includes (1) 1 sandplay sandbox, (2) 2 toy racks, (3) about 1,000 toys, (4) one digital camera used for taking pictures in the gallery, and (5) forms recording relevant data and psychological support teachers for record the characteristics of the works and the process of the works.

#### 2.2.2. Testing Process

All students completed the SAS scale before and after sandplay therapy, once a week per person. The control group did not intervene. By comparing the intervention group with the control group, the intervention effect of sandplay therapy on anxiety of the experimental group members was investigated. The specific experimental process is shown in Figure 1:

1. Preimplementation test: SAS (self-rating anxiety scale) [13] was used to screen the subjects (according to the diagnostic criteria of the self-rating anxiety scale in the behavioral medicine scale manual, the standard score of the self-rating anxiety scale ≥ 50 was taken as the standard for the diagnosis of anxiety disorders)
2. Sandplay intervention: choose a suitable venue, equipped with professional psychological instructors, test the students according to the norms of sand table play therapy, and record the relevant data of the test. The specific implementation process of sandplay therapy is shown in Figure 2:

- Choosing dry or wet sand: guiding: “Please choose dry sand or wet sand. The wet sand ratio is easier to accumulate, but it is harder and cooler.And the dry sand is softer, but less likely to build up. You can choose any kind of sand”
- Feeling sand guiding: “Close eyes and adjust breathing, feel the texture and the temperature of the sand with your hands, Feel what the sand says and let your imagination fly”
- Sandplay works: guiding: “Please put these toys in the sandbox and do whatever you want.” The subjects created freely. In this process, the subjects were not allowed to communicate with each other to avoid understanding each other's intentions, but the subjects could simply interact with the psychological teacher. Psychological teachers make simple records. If subjects do not take the initiative to communicate with psychological teachers, psychological teachers do not take the initiative to communicate with subjects
- Appreciating and experiencing works: guiding: “This is your own world, please experience the feelings this world brings to you.”
- Understanding and dialogue: having a dialogue about sandplay works, understanding the theme, content, and information about the mental state of the visitor. The last producer in the last round could have a modification opportunity, and after the production is finished. He could make some adjustments to the whole work, but he could not put toys. After the above operations, the team members and the team leader sat around the sandplay, told each other's intentions and feelings in combination with the order in which the toys were placed, and conducted an in-depth discussions. The discussion extended to the individual level. Finally, the group members jointly propositioned the sandplay works
- Photo record: the healer would take photos and record the box court works from different angles from directly below, left and right. And ask any subject in the group to choose any angle to take partial or overall photos of the work. It was up to the visitor to decide whether to demolish the work by himself or with the consultant

(3) Implement posttesting: immediately after completion, the intervention group and the control group were given SAS, and the intervention group members were asked to fill in the self-reflection questionnaire
(4) Follow-up visit: one month after the end, contact the two groups of testers and perform the SAS test again

### 2.3. Observation Index

SAS included 20 entries, each item was equivalent to a related symptom and was scored on a scale of 1 to 4. Among them, forward scoring questions were counted as 1, 2, 3, and 4 points. Reverse scoring questions were scored according to 4, 3, 2, and 1. Among them 5, 9, 13, 17, and 19 were entitled reverse in foreword score. The scoring standard was <50, indicating no anxiety. A standard score ≥ 50 and <59 was classified as mild anxiety. Standard score ≥ 60 and <69 was classified as moderate anxiety. A standard score greater than or equal to 70 indicates severe anxiety.

### 2.4. Statistical Method

SPSS 13.0 software was used for descriptive analysis and *t* test of the survey data.

## 3. Results

### 3.1. Anxiety Detection Rate

Among 350 vocational college students, 350 questionnaires had been recovered, and 336 were valid. The qualified rate of questionnaires was 96.00%. Among the 336 valid questionnaire respondents, 72 had SAS scores ≥ 50, and the incidence of anxiety symptoms was 25.00%. The incidence was 20.00% (34/170) for male students and 22.89% (38/166) for female students, with no statistically significant difference between the sexes (*P* > 0.05). Anxiety detection rate is shown in Table 2:

### 3.2. Effects of Sandplay Therapy

Since there was only 1 case with SAS score ≥ 70. It has been incorporated into the group with SAS score ranging from 60 to 59. After treatment, SAS scores of mild to moderate anxiety students in the intervention group decreased, and the difference was statistically significant. The difference before and after control group was not statistically significant. After sandplay therapy, the differences in SAS scores between the intervention group and the control group were found to be statistically significant for both mild and moderate anxiety. Comparison of SAS scores of the two groups before and after treatment is shown in Table 3:

## 4. Discussion

Mental health affects the life and study of higher vocational students. However, mental diseases have no obvious signs, so they are hidden and difficult to find. In addition, most vocational college students with mental diseases are unwilling to tell their parents and teachers, so colleges and families should pay attention to the mental health of vocational college students [14]. Sandplay therapy is an effective method to improve college students' unhealthy mental states, such as interpersonal maladjustment, anxiety, and attention deficits. Group sandplay therapy takes the group as the activity unit, and sandplay therapy in the group situation can promote interpersonal interaction, which has been proved to be effective [15]. Students in vocational colleges are in adolescence, and their physiological development has been basically mature, but their psychology is still immature, their ideas are also in the social survival of the fittest, and fair competition is constantly being tempered and tempered [16]. Due to the lack of a complete and rational understanding of the society in the process of ideological growth of vocational college students, it is inevitable for vocational college students to have anxiety in the positive, confused, wait-and-see, and even negative and dispirited psychology. The faster the social change, the stronger the anxiety [17]. The quantitative and qualitative results of group integrated sand table play therapy are analyzed by using the dynamic Jiugongge analysis technology of sand table works, which proves that group integrated sand table play therapy has certain applicability and effectiveness in improving the self-identity of higher vocational students [18].Group sandplay games refer to group members building sand tables in a common sandbox. The creation process needs to be based on certain principles and during the entire placement process. Team members are not allowed to communicate and interact in any form and play alone [19]. Group sandplay games can provide higher vocational students with a creative and free psychological space full of support from group members and help them relieve pressure [20, 21]. The context and form of the game itself can help vocational students to vent their internal psychological conflicts and psychological pressures. The projection of the sandplay table can help vocational students to understand themselves more comprehensively [22, 23]. After the tester completes the sandplay work creation, the psychological teachers should communicate with the tester. Psychological teachers should understand and record the inner world of the test taker, so as to prepare for the analysis of the psychological status of the test taker and the follow-up after the test [24, 25]. For example, when the tester places sand tools in the courtyard, the psychological teachers analyze the image on the right side and may reflect that the external world who pursues is practical and shared [26]. It is also very important for higher vocational students to follow up after receiving sandplay therapy. Schools can organize full-time teachers to carry out work to maintain the sustainability of the effect of sandplay therapy [27, 28]. Related theoretical and practical research explored the effectiveness of sandplay therapy as a psychological counseling model in colleges and universities and also verified the role of sandplay therapy in college mental health education [29, 30].

## 5. Conclusion

Research in this paper showed that among 350 subjects, 72 had SAS scores ≥ 50, and the subjects with anxiety symptoms accounted for 20.57% of the total sample. Since there was only 1 case with SAS score ≥ 70, it was incorporated into the group with SAS score ranging from 60 to 59. After treatment, SAS scores of students with mild to moderate anxiety in the intervention group decreased, and the difference was statistically significant. The difference before and after control group was not statistically significant. After sandplay therapy, the differences in SAS scores between the intervention group and the control group were found to be statistically significant for both mild and moderate anxiety.

According to the summary, the sandplay therapy is effective in promoting the mental health of college students and optimizing the mental health of college students. However, college students' mental health support should be a multichannel positive behavior, including family and school. The methods of mental health support should also be diversified. Colleges and mental health teachers should pay attention to adopting personalized methods of mental health support according to the special circumstances of college students.

## Figures and Tables

**Figure 1:** Experimental process.

**Figure 2:** The implementation process of sandplay therapy.

**Table 1:** Basic information of research object.

Groups	Gender		*x* ^2^	*P*	Age (*x* ± *s*)	*x* ^2^	*P*
	Male	Female					
Intervention group	12	24	2.145	>0.05	19.02 ± 0.39	1.251	>0.05
Control group	20	16			19.12 ± 0.28		

**Table 2:** Anxiety detection rate.

Groups		Intervention group	Control group
Gender	Male	12	20
	Female	24	16
SAS (50~59)	Students (*n*)	48	
	Rate (%)	66.67	
SAS (60~69)	Students (*n*)	20	
	Rate (%)	27.78	
SAS (>70)	Students (*n*)	4	
	Rate (%)	5.55	

**Table 3:** Comparison of SAS scores of the two groups before and after treatment.

SAS	Phase	Intervention group	Control group	*t*	*P*
50-59	Before treatment	55.35 ± 4.36	55.14 ± 4.28	1.80	>0.05
	After treatment	50.23 ± 5.47	54.87 ± 4.45	3.75	<0.05
60~69 and ≥70	Before treatment	64.86 ± 5.15	66.18 ± 5.06	1.68	>0.05
	After treatment	62.08 ± 6.32	65.75 ± 5.62	4.01	<0.05

## Data Availability

The data used to support the findings of this study are included within the article.
